The article "Fuzzy Support Tensor Product Adaptive Image Classification for the Internet of Things" was published in 2022. Journal: Comput Intell Neurosci.

# Fuzzy Support Tensor Product Adaptive Image Classification for the Internet of Things

**DOI:** 10.1155/2022/3532605

**Published:** 2022-02-22

**Authors:** Zhongrong Shi, Yun Ma, Maosheng Fu

**Affiliations:** ^1^Faculty of Electronic and Information Engineering, West Anhui University, Lu'An, Anhui 237012, China; ^2^Anhui Yongcheng Electronic and Mechanical Technology Co., Ltd.,, Lu'An, Anhui 237000, China; ^3^Faculty of Electrical and Opto-Electronic Engineering, West Anhui University, Lu'An, Anhui 237012, China

## Abstract

Computer vision is one of the hottest research directions in artificial intelligence at present, and its research goal is to give computers the ability to perceive and cognize their surroundings from a single image. Image recognition is an important research direction in the field of computer vision, which has important research significance and application value in industrial applications such as video surveillance, biometric identification, unmanned vehicles, human-computer interaction, and medical image recognition. In this article, we propose an end-to-end, pixel-to-pixel IoT-oriented fuzzy support tensor product adaptive image classification method. Considering the problem that traditional support tensor product classification methods are difficult to directly produce pixel-to-pixel classification results, the research is based on the idea of inverse convolution network design, which directly outputs dense pixel-by-pixel classification results for images to be classified of arbitrary size to achieve true end-to-end and pixel-to-pixel high-score image classification and improve the efficiency of support tensor product models for high-score image classification on a pixel-by-pixel basis. Moreover, considering that network supervised classification training using deep learning requires a large amount of labeled data as true values and obtaining a large number of labeled data sources is a difficult problem in the field of image classification, this article proposes using a large amount of unlabeled high-resolution remote sensing images for learning generic structured features through unsupervised to assist the labeled high-resolution remote sensing images for better-supervised feature extraction and classification training. By finding a balance between generic structural feature learning of images and differentiated feature learning related to the target class, the dependence of supervised classification on the number of labeled samples is reduced, and the network robustness of the support tensor product algorithm is improved under a small number of labeled training samples.

## 1. Introduction

Image recognition technology is an important research branch in the field of computer vision, which aims to identify various potential objects in images using computers to preprocess, extract features, analyze and understand them. Traditional image recognition models can be divided into two parts: excellent feature extraction methods are robust in various complex environments, while classifiers mainly consist of some shallow machine learning algorithms for predicting the classes to which the features obtained by the extractor belong. For example, in the field of face recognition, researchers can improve the accuracy of a large number of face image samples by simply feeding them to a model, which can then be trained over some time by deep learning models by more than a dozen percentage points over traditional models [1]. Excellent feature extraction methods are robust in various complex environments, while classifiers mainly consist of some shallow machine learning algorithms for predicting the classes to which the features obtained by the extractor belong. Target detection, one of the most challenging research hotspots in computer vision, is also a fundamental technique for solving more complex and advanced vision tasks such as semantic segmentation, target tracking, image description, and scene recognition. Deep learning techniques, which have emerged in recent years, are a powerful method for learning feature representations directly from data and have already brought breakthroughs in the field of target detection. Currently, the most popular image recognition techniques include image classification, target detection, target tracking, and semantic segmentation, and a huge amount of problems in computer vision can be solved perfectly using these four techniques, either directly or indirectly. These techniques assist computers in extracting, analyzing, and understanding useful information from a single or a series of images, and the trend is for deep learning models to gradually replace traditional latent recognition models. However, while various popular algorithms or models embody excellent performance, there are still some general problems and challenges, such as the insufficient number of samples, poor target viewability, and slow convergence of models to train.

The article "Fuzzy Support Tensor Product Adaptive Image Classification for the Internet of Things" was published in 2022. Journal: Comput Intell Neurosci.

With the rapid development of artificial intelligence techniques and computer performance, image recognition based on machine learning algorithms has rapidly expanded from targeted application scenarios to become a standard scientific tool and applied to the full range of natural science and technology applications. In this article, we propose a novel adaptive image classification method, the particle swarm optimized fuzzy support tensor machine [2]. The method firstly calculates the fuzzy affiliation of each sample by fuzzy affiliation function to reduce the influence of noise points on the classification results; secondly, it uses particle swarm algorithm to perform parameter search for fuzzy support tensor machine; although it is more concise and easy to operate compared with other commonly used parameter optimization algorithms such as genetic algorithm and least squares method, the particle swarm algorithm still has the disadvantage of easily falling into local optimum in this article[3]. To solve this problem, the particle swarm algorithm is improved: firstly, the inertia weights are introduced into the particle swarm algorithm, which decreases nonlinearly with the number of iterations to improve the algorithm's optimality seeking ability, and secondly, the simulated image recognition algorithm is used to make the particles in the particle swarm algorithm forcefully jump out of the local optimum trap with a certain probability. The improved particle swarm algorithm greatly improves the efficiency of the optimization search and overcomes the blindness of parameter selection in the traditional classification model.

## 2. Related Work

Unlike pixel-based classification methods, object-oriented classification methods use the segmented objects or regions of an image as the minimum unit of analysis to compensate for the lack of contextual or spatial relationships in pixel-based classification methods. Object-oriented classification methods usually use segmentation before classification and obtain the classification results of the image by extracting features from the segmented results and then training the classifier.

In the literature [4], a nonparametric Bayesian hierarchical model is proposed for high-resolution remote sensing image classification using a combination of object-oriented oversegmentation and hierarchical Dirichlet process model (HDP) and Indian buffet process (IBP), which solves a series of problems such as the traditional probabilistic topic model and ignores spatial information, and the number of topics has to be predetermined; in the literature [5], a remote sensing image is proposed for object-oriented Markov region penalty method for remote sensing images, using mean shift algorithm for image segmentation and establishing weighted region neighborhood map based on region size and neighboring region connection strength, while using region size and neighborhood strength features as penalty terms to calculate potential functions, and using maximum posterior probability to iteratively update joint probability distribution and likelihood function to obtain the final semantic segmentation results. This approach can better weigh the interactions between neighbors and obtain more macroscopic texture features; in the literature [6], after superpixel segmentation using the simple linear iterative clustering (SLIC) method, visual features are extracted and trained on the mixture components generated by the Dirichlet process mixture model through a multiple conditional random field model to obtain intermediate labels corresponding to visual features in the new feature space. Using the intermediate labels, further pixel semantic analysis is performed to establish the connection between low-level features and high-level semantics based on the spatial relationships taking into account the objects; literature [7] uses the watershed algorithm to record the process of gradual merging of oversegmented regions by region similarity comparison after oversegmenting the image using a binary segmentation tree, on which the ascending trajectory between the leaf nodes to the root node is the region evolution process obtained computationally, and the search for salient region content is achieved by finding the maximum value through first-order derivation of the evolution value, which improves the previous complex tree construction model and thus achieves image classification and target recognition more simply and efficiently. In the literature [8], a region of interest detection algorithm based on the MFF (Multiscale Feature Fusion) algorithm is proposed, which detects the region of interest in remote sensing images accurately and quickly by performing grayscale saliency analysis based on multiscale spectral residuals and directional saliency analysis based on integer wavelet transform on remote sensing images. In the literature [9], by performing Saliency Analysis of Cooccurrence Histogram (SACH) based on cooccurrence histogram for high-resolution remote sensing images and using a saliency enhancement method based on moving K-means clustering, clear region boundaries are established for the region of interest, while improving the immunity of the algorithm to noise. To reduce the computational complexity of region of interest detection for remote sensing images, the literature [10] proposes to achieve fast and efficient region of interest detection by segmenting high-resolution remote sensing images into superpixels and generating superpixel-level saliency maps using structural tensor and background contrast, and finally by superpixel-to-pixel-based saliency analysis. To extract high-quality regions of interest with clear boundaries and no background interference from remote sensing images, a GLSA (Global and Local Saliency Analysis) algorithm based on global and local saliency analysis is proposed in the literature [11] for extracting residential regions in high-resolution remote sensing images. In addition, for common features of interest in high-resolution remote sensing images, such as residential areas, airports, aircraft, and ships, a detection algorithm based on joint multi-image saliency (JMS) is proposed in the literature [12], which processes multiple multispectral remote sensing images with similar spatial structure and spectral details by jointly using the correlation information between this set of remote sensing images to simultaneously detect the features of interest in this set of multispectral remote sensing images. The literature [13] proposes a region of interest detection algorithm based on superpixel segmentation and statistical significance analysis, which detects the region of interest in remote sensing images accurately based on the final generated significance map by fusing the statistical significance feature map based on histogram statistics and the information significance feature map based on information entropy analysis. The literature [14] proposes that candidate regions containing feature targets can be predicted by supervised learning models constructed from various salient features. Then a discriminative dictionary learning classifier based on sparse coding representation can be applied to the target candidate regions to detect feature targets in the scene, which greatly reduces the computational cost of traditional search strategies. For the airport detection problem of panchromatic remote sensing images, the literature [15] proposes to use a graph-based visual saliency model to locate the salient regions in the scene and obtain a top-down saliency map by making full use of the geometric prior knowledge of the airport runway, and finally by combining these two saliency maps, to predict the location of the airport more accurately. In the literature [16], a two-layer visual saliency analysis model is proposed to extract candidate regions of airports and aircraft, and a bag-of-words model based on dense SIFT features and Hu moment features are used to characterize the invariant features of airports and aircraft, and finally, the airport and aircraft targets in remote sensing images are accurately detected by support tensor machines.

The article "Fuzzy Support Tensor Product Adaptive Image Classification for the Internet of Things" was published in 2022. Journal: Comput Intell Neurosci.

## 3. Fuzzy Support Tensor Machine Adaptive Image Classification for the Internet of Things

### 3.1. Fuzzy Support Tensor Machine Theory

Support tensor machine based on statistical learning theory relies on its excellent learning ability and powerful generalization ability to have better results in dealing with problems with a small amount of sample data and nonlinear relationship between samples. However, there are still shortcomings in the support tensor machine model. The support tensor machine works by determining the support tensor with a small number of training samples and then finding a classification surface that can divide the samples and then classify the test samples. If there are incorrect or biased samples in the training samples to determine the support tensor, the support tensor machine cannot exclude these samples because they all have the same reliability for the test samples, so it is easy to be misled by these incorrect or biased test samples and establish the wrong optimal hyperplane, resulting in a decrease in the classification accuracy of the model. The biggest difference between standard fuzzy support tensor machine and support tensor machine is that the former has one more dimension than the latter, i.e., fuzzy affiliation. Hence, the support tensor selected by the fuzzy support tensor machine is not equivalent to that selected by the support tensor machine. To address this problem, fuzzy support tensor machines introduce the concept of a fuzzy affiliation function [17]. Each training sample is assigned a corresponding fuzzy affiliation according to its influence on the prediction result, with smaller affiliations for incorrect or biased samples and larger affiliations for correct samples, by which the problem that traditional support tensor machines are easily misled by isolated points is solved and the noise immunity of the model is improved.

As the complexity of the research problem increased, the degree of state in the problem was vague and could not be accurately described by traditional exact mathematics, and fuzzy mathematics was created to have a reasonable description of the degree of state of certain factors in the problem. The discipline was introduced in the 1950s and was mainly used to study some fuzzy problems. With the rapid development of artificial intelligence technology, fuzzy mathematics has been combined with various intelligent algorithms and is widely used in various fields. A fuzzy set is a basic concept of fuzzy mathematics. In the traditional notion of set, for an individual *u* and a set A, the relationship between them is that *u* either belongs to A or does not belong to A. These two results cannot hold simultaneously [18]. The relationship between an individual and a set, if expressed by a mathematical expression, should be

(1) $$\begin{array}{c} C_{ij}=\sum_{i=1}^{n}x_{i}^{2}\sigma_{i}+x_{j}^{2}\sigma_{j}+x_{k}^{2}\sigma_{k}. \end{array}$$

The eigenfunction cannot explicitly define data as belonging to a certain state or not belonging to a certain state. In the 1960s, researchers used feature functions to express an increasing number of classical sets by representing each data in the set as a fuzzy number, such that the domain of values of fuzzy sets was extended from the set of integers {0,1} to the set of real numbers [0,1]. Since the value of the fuzzy affiliation reflects the training points, for a certain class of defined affiliations, and the parameter *j* is a measure of the extent to which the support tensor machine misclassifies the samples, combining the two becomes a measure of how correctly the support tensor machine classifies data with different affiliations. Each training sample is assigned a corresponding fuzzy affiliation according to its influence on the prediction result, with a smaller affiliation for incorrect or biased samples and a larger affiliation for correct samples. By this approach, the problem that traditional support tensor machines are easily misled by isolated points is solved, and the noise immunity of the model is improved. Transferring the processed data as input to the prediction model, the process of finding the optimal hyperplane for the classification model can be expressed mathematically as a quadratic program if the data transferred is linearly divisible.

(2) $$\begin{array}{c} E_{\text{all}}=\sum_{i=0}^{R}\left(E_{\text{contest}}\times x+Ee\times x+\varepsilon \text{free}\times x^{2}\times d_{i}^{\left(1/2\right)}\right)+\sum_{i=0}^{K}\left(4E_{e}\times x+\varepsilon \text{decay}\times x^{2}\times d_{i}^{2}\right). \end{array}$$

Minimizing *α* in the objective function yields the quadratic counterpart of the pairwise plan:

(3) $$\begin{array}{c} I\left(X;Y\right)=\frac{K\left(x,y\right)\cdot \sum_{i=1}^{n}X_{i}Y_{i}}{M\left(x\right)}\cdot \frac{x-\alpha }{\sigma }. \end{array}$$

The major difference between a standard fuzzy support tensor machine and a support tensor machine is that the former has one more dimension, i.e., fuzzy affiliation, than the latter, so the support tensor selected by fuzzy support tensor machine is not equivalent to that selected by support tensor machine. If the relationship between the factors in the problem to be solved is nonlinear and a kernel function is introduced in the solution process, then the classification problem can be expressed in mathematical form as follows:

(4) $$\begin{array}{c} H\left(x\right)=\varphi \sum_{y\in \gamma }\sum_{x\in \chi }\left[p\left(x,y\right)\cdot \;\ln\;p\left(x,y\right)+Ax+Cy\right]+\lambda . \end{array}$$

One way to represent the above diffusion tensor is to use the covariance matrix of the Gaussian distribution, which mainly describes the diffusion process of water molecules in the tissue. The statistical scatter of the two distributions is used. In this case, tensor comparisons are made by measuring the Kullback–Leibler distance between the probability distributions afterward. The symmetric version is called *J* scatter, which was proposed by Wang and Vemuri and used for tensor distance measurements. It is shown as follows:

(5) $$\begin{array}{c} M\left(x\right)=\varphi \sum_{x\in \chi }\left[p^{2}\left(x\right)\cdot \;\ln\;p\left(x\right)\right]+Ax. \end{array}$$

Although Support Tensor Machines (STM) solve the overfitting problem in traditional SVMs, the rank-weight tensor is weakly expressive and this translation leads to poorer classification accuracy. The rank-weight tensor of STM is generalized to Tucker decomposition and CP forms to obtain stronger model expressiveness. However, the CP rank-decomposition causes an exponential increase in the number of parameters in the Tucker form, which suffers from dimensional catastrophe.

The article "Fuzzy Support Tensor Product Adaptive Image Classification for the Internet of Things" was published in 2022. Journal: Comput Intell Neurosci.

### 3.2. Fuzzy Support Tensor Machine Adaptive Image Classification for the Internet of Things

Classification algorithm design has been a hot topic in the field of machine learning, pattern recognition, and computer vision. One of the most representative and successful classification algorithms is the Support Vector Machine (SVM), which has been highly successful in pattern classification by minimizing the Vapnik–Chervonenkis dimensional and structural risk. However, standard SVM models are based on vector inputs and cannot directly deal with matrices or higher-dimensional data structures, i.e., tensors, which are very common in real life. As in Figure 1, a grayscale image is a two-dimensional matrix with height and width, which is a second-order tensor, while a multispectrum has multiple spectral bands and is a third-order tensor. When high-dimensional data are fed into the SVM, a common approach is reshaping each sample into a vector. A tensor can be seen as an extension of a matrix, which in traditional signal research can be considered as an array of different dimensions depending on the object of study. However, when the training data sample size is relatively small concerning the dimensionality of the feature vectors, this can result in overfitting and lead to unsatisfactory classification performance.

The traditional image recognition model consists of two parts: feature extractor and classifier. Feature extraction methods can be classified into texture features, shape features, bag-of-words model, sparse coding, local coding, and Fisher vectors. These feature extraction extracts feature from the image and then a set of numbers or symbols are used to represent certain characteristics of the depicted object in the image and finally, these features are recognized with the help of other machine learning methods. The classical recognition methods (classifiers) are support vector machines, decision trees, adaptive enhancement, plain Bayes, and some heuristic arithmetic [19]. These classical feature representation methods have a common feature that they all require a very specialized knowledgeable researcher to carefully design the model; however, this feature makes the model deficient in two ways: firstly, the researcher needs to spend a lot of effort to design different features for different recognition tasks; secondly, the practical application requires repeated validation and parameter tuning of the model, which is very costly to optimize.

The article "Fuzzy Support Tensor Product Adaptive Image Classification for the Internet of Things" was published in 2022. Journal: Comput Intell Neurosci.

Wavelet theory is an extended version of Fourier transform theory in which a signal is decomposed into wavelets and projected onto a set of wavelet functions. This differs from the Fourier transform, which decomposes the signal into sine and cosine components. Wavelet transform theory is popular in image processing, where it decomposes the input image into a set of images with various resolutions while reducing redundancy in the image representation [20]. The parent signal components are decomposed in an extended signal variant or a shifted wavelet. Two basic properties must be satisfied for a wavelet to be considered a wavelet. The information flow used for a single-level or one-level 2D image decomposition scheme is illustrated in Figure 2.

The inverse 2D wavelet transform used to reconstruct the image involves column upsampling and filtering for each subimage using low-pass and high-pass filters. The initial source image is constructed using the low-pass filter *L* and the high-pass filter of the resulting image for row upsampling and filtering and the summation of all matrices. By examining the saliency type focusing on bottom-up, the images can be classified into two categories, spatial domain models and transform domain models, depending on whether they are transformed in the frequency domain [21]. The so-called spatial domain saliency models process the image directly in the spatial domain and thus detect the salient targets or regions of interest in the image. Therefore, in the design of saliency models, regions in the image scene with unique color features or pattern features should have high saliency, while homogeneous regions in the scene should have low saliency. Features that frequently appear in the image scene should be suppressed. Salient pixels in an image should be clustered together rather than scattered throughout the image. Therefore, the Euclidean distance in spatial location of image blocks containing contextual information about each pixel in the image is also important, because the distribution of image blocks in the background region is either far or near in space, while the distribution of image blocks in the salient target region tends to be clustered together in space. The saliency detection results can be further enhanced by incorporating the central prior knowledge of the salient regions. The saliency of pixel I in an image at a single scale can be defined as follows:

(6) $$\begin{array}{c} {P_{i,j}}^{k}\left(t\right)=\sum_{i=1,j=1}^{n,m}{\left[t_{i,j}\left(k\right)\right]}^{2}{\left[\eta_{i,j}\left(t\right)\right]}^{\beta }. \end{array}$$

Furthermore, considering that image blocks in the background region are similar at multiple scales, in contrast, image blocks in the saliency region may be similar at only a few scales but not at all scales. Therefore, multiple scales can be used to further reduce the saliency of background pixels and enhance the contrast between salient and nonsalient regions. Unlike the spatial domain saliency model, the transform domain-based saliency model requires first transforming the image from the spatial domain to the frequency domain, then processing and analyzing the image in the frequency domain, and finally obtaining the final saliency detection results by transforming the analysis results in the frequency domain back to the spatial domain. For a two-dimensional signal like an image, by performing the Fourier transform on it, the resulting image amplitude spectrum clarifies the percentage of each sinusoidal component, while the phase spectrum of the image gives the position of each sinusoidal component in the graph. In the reconstruction of the image in the Fourier transform domain, the positions located in the horizontal or vertical directions with weak periodicity or homogeneity correspond to the positions of the candidate targets in the image, and thus it is known that the saliency information of the image is implicit in the phase spectrum of the image. Therefore, the saliency detection result of the image can be obtained by extracting the phase spectrum information of the image. The initial saliency analysis results are smoothed by a two-dimensional Gaussian filtering function *g*(*x*, *y*) to obtain a visually superior final saliency map as follows:

(7) $$\begin{array}{c} e_{j}=-k\sum_{i-1}^{n}p_{i}\ln\frac{1}{p_{i}}. \end{array}$$

From the above analysis, it can be seen that the PFT transform domain saliency detection model has the advantages of simple and easy algorithm and fast operation, thus giving fast saliency detection results for a given image, but the disadvantage is that the local saliency features of the image are not considered, and it lacks suitable biological psychological support and explanation. After each iteration step, the optimization progress of the solution needs to be measured by a predefined criterion that determines whether the current state is the best fit or not. Among the saliency analysis models for natural images, the center prior and the boundary prior are the two most widely used prior knowledge, which achieves good detection results in the saliency detection of natural images, thanks to the imaging mechanism of natural images, where the salient targets of natural images are usually at the location of the image center, while the boundaries of natural images usually do not have a distribution of salient targets.

The article "Fuzzy Support Tensor Product Adaptive Image Classification for the Internet of Things" was published in 2022. Journal: Comput Intell Neurosci.

Using superpixel segmentation methods, an image is segmented into many superpixels. Each superpixel contains a large number of spatially close neighboring samples that have a similar texture, color, luminance, and other characteristics. Compared to pixel-based hyperspectral image classification methods, the superpixel-based classification methods demonstrate good regional consistency.

The superpixel segmentation process is shown in Figure 3.

To alleviate pseudoboundaries that cause misclassification, we propose a new nonlocal decision-based region delineation method. In hyperspectral images, we usually consider that the samples in local regions belong to the same class, which is local information. However, nonlocal information is also very critical in hyperspectral images. This is because samples of the same class may also be located in different regions of the image. In nonlocal decision making, pixel pair similarity is extended to superpixel pair similarity, taking into account the structural information of the current samples. For those samples that are judged to be in heterogeneous regions by the local decision, the similarity between the current sample and the filter neighborhood samples is calculated. The current sample is represented by a global search for all similar samples. Then, this similarity is compared with the calculated adaptive threshold. If the similarity of all neighborhood pixels all is greater than the threshold, the current sample is judged to be in the homogeneous region and vice versa. This model includes two stages: the first stage is to enhance the input image, then input the residual network to carry on the supervised contrast learning, and get the pretraining model; the second stage is to fix the parameters of the pretraining model and the fuzzy support tensor machine is trained to get the prediction label. In the first stage, in order to enhance the discriminative ability of feature extraction, local information, nonlocal information, and generic structured features that come from unlabeled high-resolution images are also introduced, respectively. After an image of arbitrary size is input to the network as input data, the input data are convolved by each branch in the subnet separately utilizing dense convolution operations at different scales to associate the final extracted results, reduce the dimensionality through the transition layer, and then use the output data to (1) obtain the pixel-by-pixel classification results with the classifier to compare with the reference marker to calculate the loss; and(2) input them to the next subnetwork. The above process is repeated until the final objective function is obtained. The overall loss function is calculated jointly for all the objective functions and the network is trained by backpropagation of stochastic gradient descent. To facilitate training, the weights of the objective functions of all classifiers are learned in an alternating manner with the learning of other network parameters.

The article "Fuzzy Support Tensor Product Adaptive Image Classification for the Internet of Things" was published in 2022. Journal: Comput Intell Neurosci.

## 4. Experimental Verification and Conclusions

We compare the model in this article with Single Task Learning (STL), Tensor Train Multitasking (TT-MTL), and Tucker-based multitasking models. For a fair comparison, the same network architecture is used for all methods. In all experiments, this article sets the model format to *M* = 3 and *N* = 2. Since the model is harder to train when *M*, *N* is larger because of the presence of a fifth-order tensor. (Perhaps this can be solved by trying to decompose the larger cores further.) In this article, we use this relatively lightweight structure for our experiments. For the choice of rank, the model parameters are extremely large when the rank is particularly large, so a relatively small rank (3, 4, 5) is used. The MNIST 10-class classification problem can be converted to a ten one-vs-all binary classification problem. This conversion allows the construction of a 10-task classification problem of the same kind, that is, by performing a softmax normalization on the ten classifiers before training. In this experiment, this article focuses on two performance metrics: one is the average accuracy of the ten binary classification problems, and the other is the accuracy of classifying a single digit by performing a softmax on the one-vs-all output of each task (multiclass classification accuracy). In this article, the first three convolutional layers are set to be hard-shared across all MTL models (for common feature extraction), and then the next FC layer is converted to a different multitask tensor network model format. In this article, we train with different sized subsets of the training dataset and test the model using the same test set (from 10% to 100% of the training set). As is shown in Figure 4, all MTL methods outperform STL for both more and less training data. Also, TT outperforms Tucker when the training data are small, while the results are reversed when the training data are large. The CTN proposed in this article outperforms all other methods.

The article "Fuzzy Support Tensor Product Adaptive Image Classification for the Internet of Things" was published in 2022. Journal: Comput Intell Neurosci.

In the whole experimental process, 100,000 training iterations are set in this article because the experimental images are few sample data, the choice of iteration parameters will affect the final model effect, and the accuracy and loss function of the model training can be analyzed to see in which interval the network reaches a stable equilibrium state so that the network training is in the optimal state, the accuracy and loss function curves are plotted and different network modules are designed to design the node embedding network, and the experimental results are shown in Figure 5. The comparison experiment of SE-ResNet structure and simple node embedding network access GNN can be obtained, the red line is the change curve of NSE-ResNet-EGNN network obtained by node embedding using SE-ResNet structure, and the blue is the change curve of simple node embedding network EGNN. This indicates that the extracted finite number of feature parameters can fully reflect the transient response of the actual waveform pattern. From the accuracy change curve, we can see that the two approaches are almost the same in terms of the convergence speed in the early stage, but in terms of the final convergence result, the node embedding using the SE-ResNet network model can achieve higher accuracy, and in the subsequent iterations, the trend of the network curve is smoother compared to the simple node embedding network. From the loss change curve, we can see that the node embedding using the SE-ResNet network model makes the loss function fall faster in the training process and can maintain a smoother convergence effect compared with the original knot, and from the final convergence, the node embedding using SE-ResNet network model will have less loss, and we can see that by improving the dependency relationship between node channels, the performance of the node embedding network can be effectively enhanced by improving the dependencies between the node channels.

Though the previous experiment, it can be obtained that improving the node embedding network can increase the information encoded to the nodes, thus making the edge features describe the nodes more accurately. The network design of node update is also available in the GNN-Block module, so two sets of comparison experiments are set up in this experiment from the number of Conv-Blocks in the node update network and the network architecture, respectively. To verify the effect of the number of Conv-Blocks on the final results, we choose the node update framework as the comparison experiments, whose experimental results are shown as the yellow and red curves in Figure 6, respectively. From the accuracy change curve, we can get that increasing the Conv-Block of the node update network can improve the final classification accuracy within a certain range and keep the same convergence speed in the early stage, but in the final convergence result, the number of Conv-Block is proportional to the classification accuracy within a certain range using the node update network. From the loss variation curve, we can see that as the number of Conv-Blocks of the nodal update network increases, the loss function decreases faster due to the more parameters and better robustness of the network. Regarding network depth, and from the final improvement results, increasing the complexity of the node update network can improve the few-sample classification performance within a certain range.

The article "Fuzzy Support Tensor Product Adaptive Image Classification for the Internet of Things" was published in 2022. Journal: Comput Intell Neurosci.

To visualize the effectiveness of the proposed algorithm, the distribution of representation coefficients and the corresponding normalized reconstruction residuals of the MFCARC algorithm are given. In our experiments, we selected the Indian Pines dataset for analysis, selected ten random samples from each feature class to construct the training dictionary, and randomly selected one sample from class 6 (grass/trees) of this dataset as the test book and then analyzed the representation coefficient distribution of this sample. Since the decomposition calculation process has a truncation process of redundant columns for the tensor factor matrix, some errors are inevitable while simplifying the calculation process. As shown in Figure 7, the distribution of the correlated adaptive representation coefficients based on different features exhibits the feature that the part of the representation coefficients with larger weights is mainly concentrated in the category to which the test sample belongs. From the minimum representation residual criterion, it is known that the category to which the test sample belongs should have the smallest normalized residual value by comparing the reconstruction error of the test sample and each category of dictionaries. From Figure 7, it can be found that the correlated adaptive representation models based on spectral features, DMP features, and LBP features all make correct feature category determination for the test sample, but the correlated adaptive representation model based on Gabor features incorrectly determines the sample as category 4 (maize).

The article "Fuzzy Support Tensor Product Adaptive Image Classification for the Internet of Things" was published in 2022. Journal: Comput Intell Neurosci.

Most detection models are less effective in detecting smaller objects than in detecting larger objects. This is mainly because, after multiple layers of convolution, small objects may not retain any information in the feature mapping at the topmost layer of the model. Increasing the size of the model input (e.g., from 300 × 300 to 512 × 512) can help the model improve its performance in detecting small objects, with a 2.5 percentage point improvement in mAP for SSD and a 3.2 percentage point improvement in EAO. The analysis suggests that this is related to the multiresolution detection layer proposed in this article, which gives different detection layers to detect objects of different sizes, such as the low-resolution detection layer used to improve the detection rate of small targets. The experimental results in Figure 8 are from seven smaller objects (bird, boat, chair, etc.) in PACAL_VOC2007, with XL, *L*, *M*, *S*, and XS in the horizontal coordinates denoting extra-large, large, medium, small, and very small, respectively, and the vertical coordinates denote the average detection accuracy of the model Here the different size pairs are produced by hand cropping postprocessing formation. From the figure, it can be seen that EA0 outperforms the base model SSD almost across the board and the advantage is more pronounced when the object size is of S and XS level. The analysis suggests that this is related to EA0's strategy of using different shapes and numbers of a priori frames at different detection layers and assigning more detection frames to lower resolution layers based on the results of the cluster analysis. The best results achieved by EA0 in all scales of objects also reflect the lower sensitivity and greater robustness of the model to bounding box size than SSD.

## 5. Conclusion

Deep learning has been a great success in the fields of image recognition, speech recognition, and machine translation. Among them, support tensor machines have made breakthroughs in image detection, image classification, image segmentation, face recognition, video tracking, and other vision-related domains and have achieved great success in these fields. It is due to the powerful feature extraction capability of support tensor machines in image classification that more and more scholars are applying support vector machines to image classification. Tensor algorithms have different decompositions in several scientific fields. The different decomposition methods have their own advantages and areas of application. In this article, we propose an end-to-end, pixel-to-pixel IoT-oriented fuzzy support tensor product adaptive image classification method, introduce the background of the current topic of image classification and the significance of the research, as well as the current state of research on image classification, and draw out the difficulties faced by existing image classification methods by analyzing the characteristics of image classification and the advantages and disadvantages of existing image classification, providing strong realistic implications.

The article "Fuzzy Support Tensor Product Adaptive Image Classification for the Internet of Things" was published in 2022. Journal: Comput Intell Neurosci.

The accuracy of the prediction of the classification model established using fuzzy support vector machine and the selection of parameters of the algorithm have a great relationship, the more reasonable the selection of parameters, the higher the accuracy. Therefore, in this article, to minimize the influence of parameter selection on the classification accuracy of IoT image recognition, nonlocal adaptive information is introduced, and the improved nonlocal information is combined with the fuzzy support vector machine to apply to the image classification research. This new approach to image classification is also the innovation of this paper. Experiments show that the model has better performance than standard RBMs in feature extraction and denoising tasks. Two visible and hidden layers of TRRBM are represented as matrix product states (MPS) and all computations can be done on a single kernel. This can significantly improve the computational complexity of the learning algorithm.

## Figures and Tables

**Figure 1:** Picture and tensor representation.

**Figure 2:** Wavelet decomposition of the two-dimensional image.

**Figure 3:** Superpixel segmentation process.

**Figure 4:** The average accuracy of binary classification for different algorithms with the same dataset.

**Figure 5:** Classification accuracy and loss line of the model.

**Figure 6:** Classification accuracy and loss lines of the model under different GNN-blocks.

**Figure 7:** Normalized residuals for different algorithms.

**Figure 8:** Comparison of recognition accuracy of different models for images of different sizes.

## Data Availability

The data used to support the findings of this study are available from the corresponding author upon request.

## References

[1] Smys S., Basar A., Wang H. (2020). Hybrid intrusion detection system for internet of things (IoT). *Journal of ISMAC*.

[2] Rayhana R., Xiao G., Liu Z. (2020). Internet of things empowered smart greenhouse farming. *IEEE Journal of Radio Frequency Identification*.

[3] Wang X., Gao S. (2021). A chaotic image encryption algorithm based on a counting system and the semi-tensor product. *Multimedia Tools and Applications*.

The article "Fuzzy Support Tensor Product Adaptive Image Classification for the Internet of Things" was published in 2022. Journal: Comput Intell Neurosci.

[4] Li Y., Huang Y., Zhang M., Rajabion L. (2020). Service selection mechanisms in the Internet of Things (IoT): a systematic and comprehensive study. *Cluster Computing*.

[5] Zhang J., Tao D. (2020). Empowering things with intelligence: a survey of the progress, challenges, and opportunities in artificial intelligence of things. *IEEE Internet of Things Journal*.

[6] Ruta M., Scioscia F., Loseto G. (2019). Machine learning in the Internet of Things: a semantic-enhanced approach. *Semantic Web*.

[7] Mafi M., Izquierdo W., Cabrerizo M. (2020). Survey on mixed impulse and Gaussian denoising filters. *IET Image Processing*.

[8] Wang C. (2020). IoT anomaly detection method in intelligent manufacturing industry based on trusted evaluation. *The International Journal of Advanced Manufacturing Technology*.

[9] Yacin Sikkandar M., Alrasheadi B. A., Prakash N. B., Hemalakshmi G. R., Mohanarathinam A., Shankar K. (2021). Deep learning based an automated skin lesion segmentation and intelligent classification model. *Journal of Ambient Intelligence and Humanized Computing*.

[10] Li D., Cai Z., Deng L., Yao X. (2019). IoT complex communication architecture for smart cities based on soft computing models. *Soft Computing*.

[11] Nguyen H. L., Vu D. T., Jung J. J. (2020). Knowledge graph fusion for smart systems: a Survey. *Information Fusion*.

[12] Sankaranarayanan S., Prabhakar M., Satish S., Jain P., Ramprasad A., Krishnan A. (2020). Flood prediction based on weather parameters using deep learning. *Journal of Water and Climate Change*.

[13] Sun Y., He S., Tong F. (2020). Media access control for narrowband internet of things: a survey. *Encyclopedia of Wireless Networks*.

[14] Wang P., Yang L. T., Li J., Chen J., Hu S. (2019). Data fusion in cyber-physical-social systems: state-of-the-art and perspectives. *Information Fusion*.

[15] Lau B. P. L., Marakkalage S. H., Zhou Y. (2019). A survey of data fusion in smart city applications. *Information Fusion*.

[16] Vidyashree S. (2021). Smart shopping using android application. *Journal of Research Proceedings*.

[17] Mansour R. F., Escorcia-Gutierrez J., Gamarra M., Gupta D., Castillo O., Kumar S. (2021). Unsupervised deep learning based variational autoencoder model for COVID-19 diagnosis and classification. *Pattern Recognition Letters*.

[18] Han Y., Zhang C. J., Wang L. (2019). Industrial IoT for intelligent steelmaking with converter mouth flame spectrum information processed by deep learning. *IEEE Transactions on Industrial Informatics*.

[19] Haji S. H., Sallow A. B. (2021). IoT for smart environment monitoring based on Python: a review. *Asian Journal of Research in Computer Science*.

The article "Fuzzy Support Tensor Product Adaptive Image Classification for the Internet of Things" was published in 2022. Journal: Comput Intell Neurosci.

[20] Chandra Shit R. (2020). Crowd intelligence for sustainable futuristic intelligent transportation system: a review. *Iet Intelligent Transport Systems*.

[21] Fotso Kamga G. A., Bitjoka L., Akram T., Mengue Mbom A., Rameez Naqvi S., Bouroubi Y. (2021). Advancements in satellite image classification: methodologies, techniques, approaches and applications. *International Journal of Remote Sensing*.

